The article "Integrated use of phosphorus, farmyard manure and biofertilizer improves the yield and phosphorus uptake of black gram in silt loam soil" was retracted in 2022. Reasons: compromised peer review; a conflict of interest; concerns about the authorship.

# Integrated use of phosphorus, farmyard manure and biofertilizer improves the yield and phosphorus uptake of black gram in silt loam soil

**DOI:** 10.1371/journal.pone.0266753

**Published:** 2022-04-14

**Authors:** Jagdish Singh, Rajan Bhatt, Dhaliwal S. S., B. S. Dhillon, Asma A. Al-Huqail, Alanoud Alfagham, Manzer H. Siddiqui, Hayssam M. Ali, Faheema Khan, Ritesh Kumar

**Affiliations:** 1 Punjab Agricultural University Regional Research Station, Gurdaspur, Punjab, India; 2 Punjab Agricultural University Regional Research Station, Kapurthala, Punjab, India; 3 Department of Soil Science, Punjab Agricultural University Ludhiana, Punjab, India; 4 Department of Botany and Microbiology, College of Science, King Saud University, Riyadh, Saudi Arabia; 5 Department of Agronomy, Kansas State University, Manhattan, KS, United States of America; The University of Haripur, PAKISTAN

## Abstract

An experiment on the use of farmyard manure and biofertilizer along with application of chemical phosphorus was conducted to assess the impact of differential doses of phosphorus, farmyard manure and consortium biofertilizer application on the development, yield and phosphorus uptake during the year 2018 and 2019. The impact of different treatments was recorded on the plant height, dry matter partition, yield and yield attributes, phosphorus uptake and soil phosphorus availability using standard methods. The data revealed significant improvement in yield, yield attributes, phosphorus uptake and soil phosphorus availability. The integration of farmyard manure and biofertilizer with 60 kg ha^-1^ SSP (single superphosphate) has improved the black gram yield by 7.4% and 3.28% respectively over the use of 60 SSP alone. The phosphorus uptake in black gram with application of Farm yard manure and biofertilizer along with 60 kg ha^-1^ SSP has improved the uptake by 7.18% and 2.51% respectively over the use of 60 kg ha^-1^ SSP alone. The results highlight the need of integrated application of farm yard manure, biofertilizer for sustainable production of black gram in the region.

## 1. Introduction

Black gram (*Vigna mungo* L) is a leguminous short-season crop that is one of India’s most significant pulse crops. Black gramme seeds contain 17 to 34 percent protein, making them a cost-effective source of protein. [1]. The black gram was cultivated over 3.51 million ha area and production of about 2.08 million tons, with 593 kg ha^-1^ average productivity in India in the year 2017–18 [2]. Phosphorus is a primary macronutrient, essential for plant growth and development. The earth crust contains about 0.1% phosphorus, where most of this is present either in insoluble or unavailable form to plants. The low availability of phosphorus in the soil limits about 40% of crop production in cultivated areas around the globe [3]. The problem of P unavailability further aggravates as the added P fertilizers undergo fixation at exchange complexes within the soil make it unavailable to plants [4].

Phosphorus is an essential component of nucleic acid, phospholipids, protein, coenzyme, and the energy cycle, and plays a significant role in plant growth, root development, nodulation, nitrogen fixation, flowering, and fruiting [5–7]. The addition of phosphorus improves the grain yield of legumes crops such as *Phaseolus vulgaris* [8], *Glycine max* [9], *Vicia faba* [10], *Cicer arietinum* [11], *Vigna unguiculata* [12], etc. The excessive use of phosphatic fertilizers has been associated with soil and water pollution [6], i.e eutrophication of lakes and water bodies.

The integrated use of organic manures and chemical fertilizers in crop production has proved to be helpful in maintaining higher crop productivity and sustainability in crop production [13]. The organic materials are known for their potential to act as an alternative source of multiple nutrients and their capability to improve the soil characteristics such as bulk density, water holding capacity, soil microbial activities, soil structure and infiltration rate, while reduces soil compaction and soil erosion [14, 15]. Therefore, application of phosphorus with organic manure and bio fertilizers may help in compensating the supply shortage and rising price of chemical fertilizers. Many studies have concluded that crops utilize only 15–20% of the applied phosphorus [16, 17] and remaining get fixed in soil or converted to the form not readily available to the crops [18]. Biofertilizers (*Azotobacter*, *Azospirillum*, *Rhizobium*, *phosphobacteria* and *VAM* fungi) are proving to be cost-effective alternative to expensive fertilizers, supplement nitrogen and phosphorus fertilizers by fixing environmental nitrogen, converting insoluble phosphorus from the soil into soluble form, enhances soil nutrient availability to the plants [19] and improves crop yields.

Integrated approach of nutrient management may derive maximum benefits from organic and inorganic fertilizers in an integrated manner and helps in maintaining optimum soil fertility and crop productivity [20]. Hence, the experiments under consideration were undertaken to access the response of black gram to differential doses of phosphorus, FYM and consortium biofertilizer application.

## 2. Materials and procedures

### 2.1 The soil and the experimental site

The investigation was carried out during the summer season of the year 2018 and 2019 to access the impact of unified phosphorus management on the growth, yield and phosphorus uptake in black gram. The field experiment was initiated at the farm of Punjab Agricultural University Regional Research Station, Gurdaspur, India, situated at 32.05° N and 75.43° E at an elevation of 225 m above mean sea level. The soil of the experiment site is characterized as the silt loam in texture with bulk density 1.49 Mg m^-3^, pH 7.6 (1:2 soil: water ratio), electrical conductivity of 0.20 dSm^-1^, 0.23% organic carbon, 19.0 kg ha^-1^ available phosphorus, 118.2 kg ha^-1^ available potassium.

The experimental site is characterized as subtropical and semi-arid climate and receives about 700 mm rainfall annually. The weather during the study period is characterized as hot and dry summers (April-June), where temperature ranges from 16–42° C. The mean maximum temperature recorded is as high as about 42° C in the May- June months.

### 2.2 Treatments and experimental design

Current investigation comprised of eight treatments which laid out in randomized complete block design with three replicates during both the years. The treatments include T_0_-control, T_1_-60 kg ha^-1^ SSP, T_2_- 2.5 t ha^-1^farmyard manure (FYM), T_3_-2.5 t ha^-1^ FYM + 60 kg ha^-1^ SSP, T_4_-2.5 t ha^-1^ FYM + 30 kg ha^-1^ SSP, T_5_-consortium biofertilizer, T_6_-Consortium+60 kg ha^-1^ SSP and T_7_-Consortium+30 kg ha^-1^ SSP. The whole of the nitrogen was broadcasted at the time of sowing using urea (46% N) and phosphatic fertilizer was used as per treatments through single superphosphate (16% P_2_O_5_). Each replication plot was 2.6 m wide x 3.0 m long. The well rotten farmyard manure (FYM) was added to surface soil and mixed before sowing as per treatment. The FYM had 0.58% N, 0.25% P and 0.57% K. The consortium biofertilizer consist of Phosphorus Solubilizing Bacteria, Azotobacter and Plant Growth Promoting Rhizobacteia. The powdered consortium biofertilizer was moisten and uniformly allocated over black gram seeds. The consortium biofertilizer coated seeds were air dried under shade before sowing.

### 2.3 Crop management

The sowing of black gram cultivar Mash-1008 was done in the first fortnight of the march during the year 2018 and 2019. The sown of black gram was done with row spacing of 22.5 cm with seed rate of 50 kg ha^-1^. Pendimethlin @ 2.5 liter per hectare was sprayed after sowing to check the weeds. All the fertilizers application, weed control, insect-pest control, irrigation and other cultural practices were done as per the PAU package of practices for rabi crops.

### 2.4 Soil and plant observations

In each plot, five plants were chosen at random and tagged to record observations on plant height, branches per plant, number of pods per plant, and number of seeds per pod. Dry matter partitioning was performed on a representative plant from each plot, with leaf, stem, and roots dried separately. The roots were excavated by inserting iron pipe (6 inches diameter) into the soil keeping the plant base at the centre of pipe. The soil thus excavated was washed over the wire mesh under running water and roots were separated. The leaf, stem and roots were dried in an oven at 60°C till the constant weight was achieved. The grain yield and straw yield were recorded on whole plot basis and converted into t/ha. The thousand grain weight at harvesting was also measured.

Using a colorimeter, the phosphorus content of plant tissue was measured using the vanado-molybdate method [21]. Phosphorus uptake was calculated by multiplication of P content (%) in grain with the grain yield (kg ha^-1^).

### 2.5 Analytical statistics

The data from the plants were subjected to an analysis of variance (ANOVA) using the GLM procedure in SAS 9.1 statistical software (SAS, California). The significance of differences in means was tested with the Duncan Multiple Range Test.

## 3. Results

### 3.1. Effect of different phosphorus levels, FYM and biofertilizer on plant growth and dry matter partition

The perusal of the data (Table 1) shows that the plant height was significantly affected by the application of manures, biofertilizers and phosphorus application. The data revealed that maximum plant height was observed in treatment T_3_ (18.8 cm), followed by treatment T_6_ and T_4_. At harvesting, maximum plant height was recorded in the treatment T_3_ where 2.5 t/ha FYM was applied along with 60 kg SSP, that was statistically at par with the treatment T_4_, T_6_, T_7_ and T_1_. The highest plant height under such treatment may be due to improved availability of Phosphorus and soil physical environment. The accessibility of phosphorus also improves the utilization of N and K in the plant system. As phosphorus is involved in the energy cycle of plant in addition to its involvement in protein and lipids in the plant system, that help in improving plant growth.

**Table 1:** Effect of phosphorus levels, farmyard manure and biofertilizer on plant height and dry matter accumulation.

Treatments	Plant height (cm)		Root dry matter		Leaves dry matter		Branches/stem dry matter	
	30 DAS	At harvesting	30 DAS	At harvesting	30 DAS	At harvesting	30 DAS	At harvesting
T_0_-control,	15.8c	26.1d	0.39g	2.94c	1.23g	5.31e	0.84c	4.43g
T_1_-60 kg SSP,	17.3c	30.7abc	0.53d	3.91b	1.46cd	8.31bc	0.91bc	9.54b
T_2_- farmyard Manure (FYM) 2.5 t/ha,	17.7b	29.5bc	0.43f	3.34c	1.60a	7.86c	0.93ab	5.67f
T_3_-2.5 t ha^-1^ FYM+60 kg SSP	18.8a	32.0a	0.52e	4.85a	1.44de	9.26a	0.93ab	10.04a
T_4_-2.5 t ha^-1^ FYM + 30 kg SSP	17.4b	30.7abc	0.65b	4.31b	1.53b	8.64abc	1.00a	8.33d
T_5_-consortium biofertilizer	16.4c	28.7c	0.57c	3.89b	1.50bc	6.95d	0.89b	5.31f
T_6_-consortium biofertilizer +60 kg SSP	18.5a	31.3ab	0.37h	4.29b	1.40ef	8.79ab	0.91bc	9.01c
T_7_-consortium biofertilizer +30 kg SSP	17.5b	30.1abc	0.80a	4.03b	1.37f	8.18bc	0.84c	7.22e
CV	3.22	5.68	5.57	8.30	3.20	7.96	6.28	5.30
Pr>F (Treatment)	<0.01	<0.01	<0.01	<0.01	<0.01	<0.01	<0.01	<0.01
Pr>F (Year* Treatment)	0.92	0.24	0.97	0.15	0.08	0.07	0.01	0.19
Error (MS)	0.32	2.89	0.008	0.11	0.002	0.396	0.003	0.155

The data on the root dry matter accumulation in various treatments revealed that the early root growth of black gram at 35 DAS was significantly affected by the different combinations of source of phosphorus, FYM and biofertilizers (Table 2). The root dry mass at 35 DAS (days after sowing) was higher in the treatments where chemical fertilizer were integrated with the organic and biofertilizers such as T_7_ and T_4_ as compared to application biofertilizer, organic manure and chemical fertilizer alone. The root dry matter at the harvesting stage was significantly higher in the treatment T_3_ where FYM was applied in addition to the full dose of phosphorus followed by use of biofertilizer and chemical fertilizers. Choudhary et al., [22] also reported beneficial effects of biofertilizer and organic manure on root growth and development. The recent studies had showed that phosphorus application enhanced root system resulting in better soil-root contact and finally higher P uptake and absorption of mineral nutrients [23].

**Table 2:** Yield and yield attributes under different phosphorus levels, farmyard manure, and biofertilizer treatments.

	No of pod	Grain yield (t/ha)	Biomass yield (t/ha)	Thousand grain weight (g)	Grain P content (%)
T_0_-control,	18.6c	3.54d	16.51d	37.34b	0.207a
T_1_-60 kg SSP,	25.9b	4.57ab	19.73ab	39.02a	0.215a
T_2_- farmyard manure (FYM) 2.5 t/ha,	25.9b	4.24bc	18.01c	38.14ab	0.211a
T_3_-2.5 t ha^-1^ FYM+60 kg SSP	29.7a	4.91a	20.99a	39.0a	0.215a
T_4_-2.5 t ha^-1^ FYM + 30 kg SSP	26.5b	4.55ab	19.08bc	38.12ab	0.211a
T_5_-consortium biofertilizer	21.5c	3.89cd	17.94c	37.92ab	0.209a
T_6_-consortium biofertilizer +60 kg SSP	28.9ab	4.72a	20.39ab	38.7ab	0.213a
T_7_-consortium biofertilizer +30 kg SSP	25.7b	4.12c	18.32c	37.78ab	0.209a
CV	9.57	6.67	5.53	3.10	2.78
Pr>F (treatment)	<0.01	<0.01	<0.01	0.21	0.26
Pr>F (Year* Treatment)	0.27	0.96	0.32	0.73	0.70
Error (MS)	5.89	0.083	1.09	0.70	0.0003

The leaf dry matter accumulation at 35 DAS was significantly higher in the T_2_ treatment (1.60 g per plant) followed by T_4_ (1.50 g per plant) and T_3_ (1.44 g per plant) as compared to the control and use of chemical fertilizer alone (T_1_). At harvesting stage, highest leaf dry matter was recorded in the treatmentT_3_ that was statistically similar to the treatments T_4_, T_6_ and T_7_ and significantly higher than the control and use of 60 kg SSP alone (Fig 1)

**Fig 1:** Effect of phosphorus levels, farmyard manure and biofertilizer on biomass accumulation at 35 DAS (a) and At harvesting (b). Bars represents error (MS).

The stem dry matter at 35 DAS was highest in the treatment T_4_ (FYM + 30 kg SSP) that was statistically at par with treatment T_3_ (FYM + 60 kg SSP) and T_2_ (FYM alone) (Fig 1). The branch dry matter at harvesting stage was highest (10.04 g per plant) in with the application of FYM along with 60 kg SSP (T_3_), that was statistically superior to use of 60 kg SSP alone (T_1_).

### 3.2 Effect of different phosphorus levels, FYM and biofertilizer on yield and yield attributes

The data revealed that the number of pods were significantly high (29.7) in the treatment T_3_ (FYM + 60 kg ha^-1^ SSP) as compared to T_1_ and statistically at par with the treatment T_6_. The thousand-grain weight was also higher in the treatment T_1_ and T_3_ that were statistically at par with the treatments T_2_, T_4_, T_5_, T_6_ and T_7_.

The black gram grain yield was significantly affected by the dose of phosphorus, FYM and biofertilizer application (Table 2). The black gram grain yield was significantly higher in the treatment T_3_ as compared to control, T_2_ and T_7_. The grain yield in T_3_ was 7.4 and 4.0% higher than the treatment T_1_ and T_6_. The application of FYM + 60 kg ha^-1^ SSP and biofertilizer +60 kg ha^-1^ SSP has improved the grain yield by 7.4% and 3.28% over the use of 60 SSP alone. The grain yield improvement may be resulted from the improved soil supply of phosphorus with the integrated use of FYM and biofertilizers. Apáez Barrios et al., [24] reported that the inadequate supply of phosphorus affects the photosynthetic processes as well as photosynthates supply to nodules and also adversely affect the root growth, activity and nodule formation.

The biomass yield of the black gram was increased with increasing rates of phosphorus application integrated with FYM and biofertilizers up to 60 kg ha^-1^ SSP. The biomass yield in T_3_ (20.99) significantly higher than the control and at par with the use of chemical fertilizer alone. The biomass yield with application of FYM + 60 kg SSP (T_3_) was 6.4 and 2.9% higher than the treatment T_1_ and T_6_. Thus, the integrated use of FYM +60 kg ha^-1^ SSP and biofertilizer + 60 kg ha^-1^ SSP has improved the grain yield by 6.4% and 3.34% over the use of 60 SSP (T_1_) alone. The improvement in biomass yield may be ascribed to the favourable effect of phosphorus application and other organics on plant height, dry matter production, and number of pods as reported by Niraj and Ved [25] and Parashar et al [26].

The grain P content was not significantly affected by the application of phosphorus, FYM and biofertilizers, however grain P content in T_3_ treatment was 3.86% higher than the control.

### 3.3 Phosphorus availability and uptake under different phosphorus levels, FYM and biofertilizer application

The data revealed highest available soil phosphorus in the treatment T_3_ followed by T_4_ and T_2_ (Fig 2B). The soil available phosphorus was highest where FYM was applied along with chemical phosphorus fertilizer. The higher soil available phosphorus in the treatments where FYM was applied may be due to addition of extra phosphorus through the FYM and decomposition of FYM produces organic acids which might had improved the availability of phosphorus in the soil. The biofertilizers has also improved the P availability due to phosphorus solubilizing action of bacteria’s and fungi applied to the seeds.

**Fig 2:** (a) Phosphorus uptake under different treatments (Bars represents standard error) (LSD = 1.92) 2 (b) Soil available phosphorus under different treatments before harvesting.

The soil availability has affected the phosphorus uptake of black grams (Fig 2A). A significantly higher P uptake was observed in the treatment T_3_ (26.4 kg/ha) as compared to control. The phosphorus uptake in treatment with application of FYM along with 60 kg ha^-1^ SSP (T_3_) was statistically at par with treatment T_6_ and T_1_. The improved soil availability may be resulted from the application of fertilizer, whereas application of fertilizer along with FYM and biofertilizer was more efficient in raising the soil available phosphorus. The microbes from the biofertilizer and organic acids from the FYM decomposition converts unavailable phosphorus to available form.

## 4. Discussion

Phosphorus plays important role in metabolic processes associated with shooting organs, energy generation, synthesis of nucleic acid, photosynthesis, and respiration of legume crops [27–29]. The P have crucial role in nodule energetic transformations thus legumes require more phosphorus as compared to cereals [30]. Phosphorus is found in soil as primary P minerals (apatite) and secondary clay minerals, such as calcium, iron, and aluminium phosphates, which are important in maintaining phosphorus buildup and availability through desorption and dissolution processes [31]. With the application of farmyard manure and biofertilizer, the field experiment revealed an increase in plant height, number of pods, root and shoot biomass, and root and shoot biomass (Tables 1 and 2). The integrated application of organics and fertilizers has increased the thousand grain weight by enhancing flowering and seed formation [32, 33]. The farmyard manure releases phosphorus and other macro and micronutrients upon decomposition, in addition it dissolves the unavailable form of phosphorus through the release of organic acids on decomposition of farmyard manures [31]. The improved availability of phosphorus in soil has been observed (Fig 2B) in response to application of farmyard manure and biofertilizer. The magnitude of availability was higher in the plots with addition of farmyard manures as compared to initial phosphorus status in the soil. The use of biofertilizers has also improved the phosphorus availability to plants due to the mineralization, solubilization and translocation action of phosphorus solubilizing through production of organic acid and proton extrusion [34, 35]. Nahas [36] attributed increase in solubilization of insoluble phosphate due to organic acids produced by microbes to the drop in soil pH, soil cations chelating, and competition with phosphate for adsorption sites in the soil solution. The increased availability of phosphorus in soil has also resulted in the improvement in phosphorus uptake in black gram (Table 2). Ganesan [37] also reported improved root and shoot growth of plant along with increased P uptake in black gram compared to untreated plants. Kaur and Reddy [38] and Shahzad et al. [39] also observed improved soil P status and plant P nutrition with inoculation with phosphate solubilizing bacteria resulted from higher alkaline phosphatase activity. Khatkar et al [40] also observed yield improvement with microbial inclulation of urdbean seeds. Thus, addition of farmyard manure not only add up to nutrient pools but also creates favourable root zone environment for better root activity and nutrient uptake. Likewise, inoculation of black gram seed with consortium biofertilizer improves soil phosphorus availability and plant uptake. Mahanta et al [41] reported inoculation of soyabean seed with phosphorus solublizing bacteria and VAM may substitute about 50% phosphatic fertilizer under soyabean-wheat crop rotation, similar results have been found with black gram in the present study.

## 5. Conclusions

The results revealed significant improvement in yield, soil phosphorus availability and phosphorus uptake in black gram. The integrated use of organic sources such as farm yard manure and consortium biofertilizers improved the phosphorus availability and uptake. The use of farm yard manure and biofertilizer in combination with 60 kg ha^-1^ SSP increased grain output by 7.4% and 3.28%, respectively, above the use of 60 kg ha^-1^ SSP alone. Thus, combined use of organic and inorganic chemical fertilizers may be recommended instead of chemical fertilizer alone to reduce the dependence on chemical fertilizers, to have improvement in soil health for sustainable production of black grams in the region.
